RETRACTED

# The Value of Combined Application of Oxycodone Hydrochloride Injection and Dexmedetomidine in Anesthesia for LC for Patients with Gallbladder Lesions

**DOI:** 10.1155/2021/1290650

**Published:** 2021-09-02

**Authors:** Zhantian Wang, Xiaofeng Xu

**Affiliations:** Department of Anaesthesiology, Second Affiliated Hospital of Xiamen Medical College, Fujian, Xiamen, China

## Abstract

**Objective:**

To analyze the effect of combined application of oxycodone hydrochloride injection and dexmedetomidine in anesthesia for laparoscopic cholecystectomy (LC) for patients with gallbladder lesions.

**Method:**

93 patients with gallbladder lesions in our hospital were divided into 2 groups by the random number table method. 46 patients in the control group applied oxycodone hydrochloride injection in anesthesia, and 47 patients in the observation group applied oxycodone hydrochloride injection combined with dexmedetomidine in anesthesia.

**Result:**

The T1 and T2 MAP levels in the observation group were lower than those in the control group (*P* < 0.05), and the difference between T3 and the control group was not significantly significant (*P* > 0.05). The T1 to T3 HR level in the observation group were lower than those in the control group (*P* < 0.05). The rate of excessive sedation (10.64%) and sedation inefficiency (12.77%) in the observation group was lower than that in the control group (28.26% and 30.43%), and the rate of satisfactory sedation (76.60%) was higher than that in the control group (41.30%) (*P* < 0.05). The postoperative awakening, tracheal tube removal, and first anal venting time were shorter in the observation group than in the control group (*P* < 0.05). The WHO scores of incisional pain at 6, 12, 24, and 48 hours after the operation were lower in the observation group than in the control group (*P* < 0.05). The T2 SOD level in the observation group was higher than that in the control group, and the ROS and MDA levels were lower than those in the control group (*P* < 0.05). The incidence of side effects of anesthetic in the observation group was 17.02%, which was not statistically different from the control group of 13.04% (*P* > 0.05).

**Conclusion:**

The combined application of oxycodone hydrochloride injection and dexmedetomidine in anesthesia for LC for patients with gallbladder lesions can achieve better sedation and analgesia effect, accelerate postoperative awakening and recovery, and control oxidative stress and fluctuations in signs, without increasing anesthesia-related side effects.

## 1. Preface

The gallbladder is the main organ that stores bile outside the liver. It is an important immune and digestive organ of the body. The main functions of the body are to shrink the gallbladder, concentrate bile, and store bile. It can be seen that the gallbladder is important for the overall maintenance of the body system [1]. Affected by changes in people's lifestyle and diet, the incidence of gallbladder lesions is gradually increasing. The treatment for gallbladder lesions can be divided into nonsurgical method and surgical method. Although nonsurgical treatment does not cause trauma, it is difficult to achieve a radical cure. The risk of later recurrence is high [2, 3].

RETRACTED

In order to ensure the completeness of the treatment, the clinical treatment of patients with surgical indications uses surgical method. Cholecystectomy is a common method for clinical treatment of gallbladder lesions. This surgical method includes traditional open cholecystectomy and laparoscopic cholecystectomy. Open cholecystectomy can directly remove the diseased tissue under direct vision. The operation accuracy is high and the effectiveness is guaranteed. However, the incision is large, the trauma is obvious, the postoperative recovery takes a long time, and the incidence of postoperative complications is high [4, 5]. With the deepening of the concept of minimally invasive surgery, laparoscopic surgery has been more and more widely used in surgical treatment. LC has mild trauma, high safety, rapid postoperative recovery, and higher acceptance by doctors and patients [6]. However, LC is essentially a traumatic operation. In order to ensure the smooth progress of the operation and improve the safety, it is very important to perform surgical anesthesia. Dexmedetomidine has an outstanding analgesic effect, which can effectively inhibit the formation of sympathetic activity and maintain cardiovascular stability [7]. Oxycodone hydrochloride injection mainly exerts its effect on smooth muscle and central nervous system and can quickly exert its effect after administration, with satisfied safety [8].

The above two drugs have been used in abdominal surgery, and studies have shown that the sedative efficiency of dexmedetomidine in gastric cancer surgery can exceed 90% [9]. Research on the application of oxycodone hydrochloride injection in the anesthesia of gallstone surgery can effectively reduce the adverse reactions of anesthesia [10]. However, there is a lack of research on the combined application of two drugs for LC surgery anesthesia. Based on this, this study selected 93 LC surgery patients in our hospital for specific analysis, and the summary is as follows.

## 2. Information and Method

### 2.1. Information

A total of 93 patients with gallbladder disease in our hospital from January 2019 to December 2019 were divided into control group and observation group, 46 cases and 47 cases, respectively. Inclusion criteria were as follows: (1) a clear diagnosis result of gallbladder disease; (2) only one type of disease appearing; (3) laparoscopic cholecystectomy performed electively; (4) American Society of Anesthesiologists (ASA) [11] grades I-II; (5) good body tolerance and ability to adapt to the operation; (6) patients signing the informed consent form for the study and the consent form for anesthesia and surgery; and (7) passing the ethical approval of the hospital. Exclusion criteria were as follows: (1) Patients have received radiotherapy before undergoing surgery. (2) Patients have complicated with immune diseases. (3) Patients have allergic reactions to opioids. (4) Patients had severe infections and malignant tumors.

RETRACTED

### 2.2. Method

After entering the room, the two groups of patients were connected to the ECG monitor and the depth of anesthesia monitor to monitor the ECG and Cerebral State Index (CSI). At the same time, noninvasive blood pressure and pulse oximetry should be monitored.

In the observation group, oxycodone hydrochloride injection combined with dexmedetomidine was used in anesthesia, and 0.04 mg/kg oxycodone hydrochloride injection and 0.5 *μ*g/kg dexmedetomidine were selected for intravenous injection before the start of the operation. Other medications included half an hour before surgery, and 0.5 mg atropine and 10 mg diazepam were injected intramuscularly. For induction of anesthesia, 0.5 mg/kg atracurium, 0.05 mg/kg midazolam, 0.4 *μ*g/kg sufentanil, and 0.2 mg/kg etomidate were used to make a rapid induction of airway intubation. After connecting anesthesia machine, mechanical ventilation was implemented, the tidal volume at 7-8 ml/kg was controlled, the ventilation frequency was maintained at 13 times/min, and the End-tidal Carbon Dioxide Partial Pressure (PetCO_2_) was controlled at (40 ± 5) mmHg. For anesthesia maintenance, 5 mg/(kg·h) propofol and 0.1–0.5 *μ*g/(kg·min) remifentanil were selected.

In the control group, oxycodone hydrochloride injection was used in anesthesia, and 0.04 mg/kg oxycodone hydrochloride injection was selected for intravenous injection before the operation. Anesthesia was maintained with 5 mg/(kg·h) propofol and 0.1–0.5 *μ*g/(kg·min) remifentanil, and CSI was maintained at 47–53. The preoperative medication, medication for induction of anesthesia, and related operations and treatments were the same as those in the observation group.

### 2.3. Observed Indicators

Heart rate (HR) and mean arterial pressure (MAP) were measured at four time points before induction of anesthesia (T0), 2 min before extubation (T1), 2 min after extubation (T2), and 5 min after extubation (T3) in both groups, respectively. HR, systolic pressure, and diastolic pressure were measured using a sphygmomanometer, and MAP = (systolic pressure + 2 × diastolic pressure)/3 was calculated.

RETRACTED

#### 2.3.1. Sedation Effect

Sedation effect was evaluated using the Riker sedation-agitation scale [12], with a score between 1 and 7. 1 is unable to wake up and completely unable to communicate with the patient. 2 is very sedated, with a slight response to somatic stimuli. 3 is sedated, with verbal stimuli that allow simple obedience to commands, while allowing rapid sleep. 4 is quiet and cooperative, with patients who can obey commands and are easy to wake up. 5 is agitated, with verbal cues that allow them to remain quiet. 6 is very agitated, requiring protective restraint. 7 is extremely agitated, and restraint is useless, showing aggressive resistance behavior. 1–2 points indicate excessive sedation, 3–4 points indicate satisfactory sedation, and 5–7 points indicate ineffective sedation and need to increase the use of sedative drugs.

#### 2.3.2. Recovery from Anesthesia

The time of postoperative awakening, time of tracheal tube removal, and time of first postoperative anal discharge were compared between the two groups. The postoperative awakening time was the interval between the cessation of anesthesia and the call for eye opening. The time of tracheal tube removal was the interval between the cessation of anesthesia and the removal of the tracheal tube. The time of first postoperative anal venting was the interval from the completion of surgical suturing until the patient's first act of anal venting.

#### 2.3.3. The Degree of Incisional Pain

The degree of incisional pain of patients was evaluated using the World Health Organization (WTO) pain grading criteria [13] at 6, 12, 24, and 48 hours after the end of surgery, respectively, and was divided into 0–IV degrees. Degree 0 means no pain. Degree I means mild intermittent pain and no medication required. Degree II means moderate continuous pain, rest disturbed, and small amount of pain medication required. Degree III means severe continuous pain and pain must be relieved with the help of medication. Degree IV means persistent severe pain, with changes in blood pressure and pulse level. The corresponding score is 0–4, with higher scores indicating more severe pain.

#### 2.3.4. Oxidative Stress

5 ml of peripheral blood was used as specimens before induction of anesthesia (T1) and during awakening from anesthesia (T2). Specimens were centrifuged at 3000 rpm for 8 mins, and serum was collected and measured by radioimmunoprecipitation kit for the level of superoxide dismutase (SOD), reactive oxygen species (ROS), and malondialdehyde (MDA).

RETRACTED

#### 2.3.5. Side Effects of Anesthesia

The perioperative nausea and vomiting, bradycardia, hypotension, drowsiness, respiratory depression, and agitation during the awakening period were compared between the two groups.

### 2.4. Statistical Method

Statistical analysis was performed with SPSS 23.0, with count data expressed as [*n*(%)]. *X*^2^ test and measurement data were expressed as ($\bar{x}$ ± *s*). *t*-test, multipoint comparison was performed with ANVOA analysis. *F*-test and graphs were produced with GraphPad Prism 8. *P* < 0.05 was considered statistically significant.

## 3. Result

### 3.1. General Information

There was no statistical difference in the proportions of males and females, the proportions of ASA grade I and grade II, and the proportions of disease types between the observation group and the control group (*P* > 0.05); and there was no statistical difference in the mean age, mean body mass, and mean operation time between the observation group and the control group (*P* > 0.05) (Table 1, Figure 1).

### 3.2. HR and MAP

There was no statistical difference in the HR and MAP level between the observation group and the control group at the time point of T0 (*P* > 0.05). The difference in MAP level of the observation group from T1 to T3 and T0 was not statistically significant (*P* > 0.05). The T1 and T2 MAP levels of the control group were higher than that of T0 (*P* < 0.05), and the T3 MAP level was not statistically different from that of T0 (*P* > 0.05). The T1 and T2 MAP levels were lower than those of the control group (*P* < 0.05), and the difference between T3 and the control group was not significant (*P* > 0.05). There was no statistically significant difference between T1 to T3 HR levels and T0 in the observation group (*P* > 0.05). T1 to T3 HR levels were significantly higher than that of T0 in the control group (*P* < 0.05), and T1 to T3 HR levels were all lower in the observation group than in the control group (*P* < 0.05) (Figure 2).

### 3.3. Sedation Effect

The rate of excessive sedation after combined application of oxycodone hydrochloride injection and dexmedetomidine in anesthesia in the observation group was lower than that in the control group with single application of oxycodone hydrochloride injection. The rate of satisfactory sedation in the observation group was higher than that in the control group, and the rate of ineffective sedation was lower than that in the control group. All difference was statistically significant (*P* < 0.05) (Table 2).

### 3.4. Recovery from Anesthesia

The postoperative awakening time was (11.24 ± 3.62) min in the observation group and (18.94 ± 5.67) min in the control group. The postoperative tracheal tube removal time was (15.42 ± 5.19) min in the observation group and (22.61 ± 7.34) min in the control group. The time for the first postoperative anal discharge was (40.61 ± 10.43) h, and that of the control group was (53.67 ± 13.49) h. The postoperative time to awaken, time to remove the tracheal tube, and time to first anal discharge were shorter in the observation group than in the control group, and the difference was statistically significant (*P* < 0.05) (Figure 3).

RETRACTED

### 3.5. Pain Degree of Incision

In the observation group, the intragroup comparison of WHO scores of incisional pain level gradually decreased at 6, 12, 24, and 48 hours after the end of surgery, and the difference in scores between different times was statistically significant (*P* < 0.05). In the control group, the intragroup comparison of WHO scores of incisional pain level gradually decreased at 6, 12, 24, and 48 hours after the end of surgery, and the difference in scores between different times was statistically significant (*P* < 0.05). The WHO scores of incisional pain degree at 6, 12, 24, and 48 hours after the end of surgery were lower in the observation group than in the control group (*P* < 0.05) (Figure 4).

### 3.6. Oxidative Stress

There was no significant difference in SOD, ROS, and MDA level between the observation group and the control group at T1 time point (*P* > 0.05). At T2, the SOD level of both groups decreased, and the ROS and MDA level increased; and the difference was statistically significant when compared with the T1 time point in the group (*P* < 0.05). SOD level at T2 time point in the observation group was higher than that in the control group, and ROS and MDA levels were lower than those in the control group (*P* < 0.05) (Figure 5).

### 3.7. Side Effect of Anesthesia

In the observation group, there were 8 patients who developed anesthetic side effect after the combined application of oxycodone hydrochloride injection and dexmedetomidine in anesthesia, and the incidence of anesthetic side effect was 17.02%. Meanwhile, in the control group, there were 6 patients who developed anesthetic side effect after the single application of oxycodone hydrochloride injection in anesthesia, and the incidence of anesthetic side effect was 13.04%. There was no statistical difference in the incidence of anesthetic side effect between the two groups (*P* > 0.05) (Table 3).

## 4. Discussion

Cholecystectomy is an effective clinical treatment for a variety of gallbladder lesions. Although the LC effectively compensates for the shortcomings of open surgery and is widely used in the clinic, the intraoperation will still form a pull on the internal organs and tissues, leading to an inflammatory response in the organism, and patients will have relatively obvious pain after surgery. In order to maximize the smooth implementation of the procedure and the patient's smooth recovery after surgery, the anesthesia method must be chosen reasonably [14].

RETRACTED

In this study, the MAP and HR levels of T1 to T3 time points in the observation group did not show significant fluctuations compared with T0. Meanwhile, the MAP levels of T1 and T2 in the control group were higher than T0, and the HR levels of T1 to T3 were higher than T0, indicating that the perioperative sign level in the control group fluctuated more significantly compared with the observation group. The sign level in the observation group was maintained at stable level during the perioperative period, while the fluctuation of sign level in the control group may have an adverse effect on the safety of surgery. The better effect of the observation group was the fact that the combined application of dexmedetomidine could significantly reduce sympathetic tone, and patients felt less pain during the perioperative period, and the stress response of the body was lighter; thus the levels of MAP, HR, and other signs did not fluctuate significantly. From the evaluation of the sedation effect, the satisfactory rate of sedation in the observation group was higher than that in the control group, and the oversedation and ineffective sedation were lower than those in the control group, indicating that the drugs applied in the observation group could obtain better anesthetic sedation and ensure the smoothness of the operation. Moreover, the incidence of anesthesia-related side effect in the observation group was not significantly different from that in the control group, indicating that the increased use of dexmedetomidine did not significantly affect the safety of anesthesia. The study showed that the sedation efficiency of the group in which dexmedetomidine was applied in combination with anesthesia was 89%, which was higher than that of the control group, 72%, which is consistent with the results of this study [15]. Compared to the control group, patients in the observation group in this study awoke earlier after surgery, had their tracheal tubes removed sooner, and also started anal venting earlier, suggesting that the recovery rate in the observation group was better than that in the control group after surgery. The reason is that the combination of oxycodone hydrochloride injection and dexmedetomidine used in anesthesia can have a synergistic effect through the exertion of their respective mechanisms of action, thus obtaining better result than that when using one drug alone. Similar studies have also shown that the combined application of dexmedetomidine in anesthesia shortens the postoperative awakening time and extubation time compared to conventional anesthesia [16].

RETRACTED

In terms of postoperative incisional pain level, the pain level was lower in the observation group at 6, 12, 24, and 48 hours postoperatively, suggesting that a more satisfactory postoperative analgesic effect could be obtained in the observation group with the drug method than in the control group. The study also showed that the pain scores were lower in the dexmedetomidine group than in the control group from 2 to 24 hours postoperatively [17], which is related to the synergistic effect of the two drugs. Dexmedetomidine, a class of *α*2-adrenoceptor agonists, can provide analgesia along with sedation and control the degree of sympathetic excitation [18]. Oxycodone hydrochloride injection is a class of dual agonists, a semisynthetic opioid, which not only has a significant analgesic effect but also does not cause respiratory depression [19]. Simultaneous application of two drugs with analgesic effect can achieve better analgesic effect. Perioperative hemodynamic changes generate more oxygen radicals, which can damage tissues after oxidation reactions with lipids in tissues, producing MDA [20]. SOD is a very important class of antioxidant enzymes in the body, which can scavenge oxygen radicals by catalytic reduction reactions [21]. In this study, SOD level decreased in both the observation group and the control group at the T2 time point compared with T1, and ROS and MDA levels increased compared with T1. However, the changes in the observation group were smaller compared with the control group, indicating that the drug administration method of the observation group could control the perioperative oxidative stress in the body. The operation in LC surgery activates the oxidative stress response and reduces the antioxidant capacity of the body. The already-existing oxidative stress can be further enhanced if patients are agitated during the postoperative awakening period [22]. The combined application of oxycodone hydrochloride injection and dexmedetomidine in anesthesia can reduce the production of oxidative products and enhance the antioxidant capacity, which can control the degree of oxidative stress [23]. The combined application of dexmedetomidine in the observation group could bind to *α*2-AR in the blue spot of the brainstem and inhibit neuronal norepinephrine release, blocking sympathetic downward conduction and reducing the amount of epinephrine release, which is one of the reasons for the milder oxidative stress in the observation group [24, 25].

RETRACTED

In conclusion, the combined application of oxycodone hydrochloride injection and dexmedetomidine in LC anesthesia for patients with gallbladder lesions can achieve better sedation and analgesia, accelerate postoperative awakening and recovery, and control the degree of oxidative stress and fluctuations in signs, without increasing anesthesia-related side effect. However, fewer subjects were included in this study, and the analysis on the mechanism of action of the combined application of oxycodone hydrochloride injection and dexmedetomidine was not in-depth enough; and only a controlled analysis of two groups was conducted, resulting in the obtained results being of poor scientific validity. In the future, more in-depth studies with larger subjects and more aspects should be conducted to obtain more scientific and representative findings.

## Figures and Tables

**Figure 1:** Age, body mass, and operative time. Compared with the control group, there was no significant difference in the observation group in terms of age (*P* > 0.05), body mass (*P* > 0.05), and operative time (*P* > 0.05).

**Figure 2:** MAP and HR. Compared to the T0 MAP (a) and HR (b) level in the control group, there was no significant difference in the observation group (*P* > 0.05). Compared with the T1 and T2 MAP (a) and HR (b) level in the control group, the observation group was lower (*P* < 0.05). Compared with the T3 MAP (a) level in the control group, the observation group was not significantly different (*P* > 0.05). Compared with the T3 HR (b) level in the control group, the observation group was lower (*P* < 0.05). ^*∗*^indicates *P* < 0.05 for the comparison between the two groups.

**Figure 3:** Time to awaken, extubation, and anal venting. Compared with the postoperative awakening time (a), time to extubation (b), and time to first anal venting (c) in the control group, all were shorter in the observation group (*P* < 0.05). ^*∗*^indicates *P* < 0.05 for the comparison of the two groups.

**Figure 4:** Postoperative pain degree of incision compared with the WHO score of incisional pain degree at 6, 12, 24, and 48 hours postoperatively in the control group; it was lower in the observation group (*P* < 0.05). ^*∗*^indicates *P* < 0.05 for comparison between the two groups.

**Figure 5:** Oxidative stress. Compared with the control group's T1 SOD (a), ROS (b), and MDA (c) levels, there was no significant difference in the observation group (*P* > 0.05). Compared with the control group's T2 SOD (a) level, the observation group was higher (*P* < 0.05). Compared with the control group's T2 ROS (b) and MDA (c) levels, the observation group was lower (*P* < 0.05). ^*∗*^indicates *P* < 0.05 for the comparison of the two groups.

RETRACTED

**Table 1:** Comparison of general information between the 2 groups ($\bar{x}$ ± *s*)/[*n*(%)].

Information	Observation group (*n* = 47)	Control group (*n* = 46)	*t/X* ^2^	*P*
*Gender*				
Male	26 (55.32)	27 (58.70)	0.108	0.742
Female	21 (44.68)	19 (41.30)		

Age (years)	56.83 ± 11.49	58.41 ± 10.92	0.679	0.499
Body mass (kg)	65.43 ± 4.92	66.91 ± 5.41	1.381	0.171
Surgery time (min)	216.35 ± 25.94	220.67 ± 23.79	0.837	0.405

*ASA classification*				
Grade I	27 (57.45)	28 (60.87)	0.113	0.737
Class II	20 (42.56)	18 (39.13)		

*Disease type*				
Gallbladder stones	15 (31.91)	15 (32.61)	0.619	0.274
Cholecystitis	13 (27.66)	14 (30.43)		
Gallbladder polyps	19 (40.43)	17 (36.96)		

**Table 2:** Comparison of sedation effect after anesthesia between two groups [*n*(%)].

Grouping	Oversedation	Sedation satisfaction	Sedation is ineffective
Observation group (*n* = 47)	5 (10.64)	36 (76.60)	6 (12.77)
Control group (*n* = 46)	13 (28.26)	19 (41.30)	14 (30.43)
*X* ^2^	4.625	11.982	4.299
*P*	0.032	0.001	0.038

**Table 3:** Comparison of the incidence of anesthesia-related side effect between the two groups [*n*(%)].

Grouping	Nausea and vomiting	Bradycardia	Low blood pressure	Drowsiness	Respiratory depression	Restlessness during the awakening period	Total incidence
Observation group (*n* = 47)	2 (4.26)	2 (4.26)	1 (2.13)	1 (2.13)	1 (2.13)	1 (2.13)	8 (17.02)
Control group (*n* = 46)	1 (2.17)	1 (2.17)	1 (2.17)	0 (0.00)	0 (0.00)	2 (4.35)	6 (13.04)
*X* ^2^							0.288
*P*							0.592

## Data Availability

The data used to support the findings of this study are included within the article.
